The article "Fibroblast Growth Factor 3 Is Associated with Tongue Squamous Cell Carcinoma: A Controlled Study" was retracted in 2023. Reasons: signs of a paper mill; suspected computer-generated content; unreliable results or conclusions; concerns about the data.

# Fibroblast Growth Factor 3 Is Associated with Tongue Squamous Cell Carcinoma: A Controlled Study

**DOI:** 10.1155/2022/3331119

**Published:** 2022-06-08

**Authors:** Yang Zhang, Pan Liu, Weipeng Su, Gaowa Aodeng, Huarong Zhao

**Affiliations:** Cancer Center, The First Affiliated Hospital of Xinjiang Medical University, Urumqi 830054, China

## Abstract

**Objective:**

To explore the effects of fibroblast growth factor 3 (FGF3) on the proliferation, cell cycle, and apoptosis of the tongue squamous cell carcinoma SCC-9 cell line (SCC-9).

**Methods:**

We measured the proliferation of SCC-9 cells in a control group, an FGF3 intervention group, and a fibroblast growth factor (FGFR) inhibitor intervention group in cholecystokinin octapeptide (CCK-8) experiments. We studied effects of FGF3 on the cell cycle and apoptosis of tongue cancer cells using flow cytometry. We further explored the IRS1/PI3K/AKT signaling pathway by measuring BCL-2 and Bcl-2 Associated X-protein (BAX) mRNA and protein levels with RT-PCR and western blot, respectively.

**Results:**

Results from the CCK-8 experiment showed that survival rates of cells in the control group, FGF3 intervention group, and FGFR inhibitor intervention group were 100.000% ± 4.026%, 136.330% ± 9.779%, and 83.199% ± 4.954%, respectively; survival rates of SCC-9 cells in all three groups were statistically significant (*P* < 0.05). Compared with that in the control group, the ratio of cells in G0/G1 phase in the FGFR inhibitor intervention group was higher (*P* < 0.05) and that in G2/M phase was lower, while the FGF3 intervention group showed opposite results (*P* < 0.05). The apoptosis rate of tongue cancer cells differed significantly between the FGFR inhibitor intervention and the control groups (*P* < 0.05). The mRNA and protein expression levels of IRS1, PI3K, and BCL-2 were all increased in the FGF3 intervention group (*P* < 0.05), while BAX mRNA and protein expression levels were decreased (*P* < 0.05). The mRNA expression levels of protein kinase B (AKT) showed no differences between groups. The p-AKT protein was overexpressed, while the total amount of AKT protein remained stable (*P* < 0.05).

**Conclusion:**

FGF3 contributes to the proliferation of SCC-9 cells by increasing the proportion of cells in G2/M phase. Therefore, appropriately timed inhibition of FGF3 can potentially promote tumor apoptosis through the IRS1/PI3K/AKT signaling pathway. Our results demonstrate the role of FGF3 in the tumor microenvironment in tongue squamous cell carcinoma SCC-9 cells and suggest new therapeutic targets.

## 1. Introduction

Tongue squamous cell carcinoma is the most common type of head and neck malignancy, and patients have poor prognosis. Patients with tongue squamous cell carcinoma are prone to tumor recurrence and metastasis, affecting the quality of life [1, 2]. Therefore, there is therapeutic interest in finding genes that influence the proliferation and apoptosis of tongue squamous cell carcinoma. Fibroblast growth factors (FGFs) are a class of protein polypeptides that are structurally related and encoded by the FGF gene family [3]. Many studies have confirmed that FGFs are highly expressed in a variety of tumors, such as lung cancer [4, 5], gastric cancer [6], and breast cancer [7], and promote tumor progression. However, few studies have reported the role of FGFs in cell carcinoma [8]. Here, we detected FGF3 in 40 cases of tongue squamous cell carcinoma and corresponding adjacent tissues by immunohistochemistry and found high expression levels of FGF3 were 90% in tumors and 12.5% in the surrounding tissues (*P* < 0.01). That proves FGF3 is significantly higher in tongue cancer relative to adjacent tissues. A variety of intracellular biological processes are regulated through the PI3K/AKT signaling pathway, including cell proliferation, apoptosis, migration, and growth; all of these processes are closely related to tumorigenesis. The present study is aimed at exploring effects of FGF3 on tongue squamous cell carcinoma and at understanding the role of FGF3 in the development of the disease in order to propose new targets for the diagnosis and treatment of oral malignant tumors.

## 2. Materials and Methods

### 2.1. Materials

The human tongue squamous cell carcinoma cell SCC-9 was purchased from Shanghai Yaji Biotechnology Co., Ltd.; fetal bovine serum (FBS) from Shanghai Ikesai Biological Products Co., Ltd.; CCK-8 cell proliferation/toxicity detection kit from Beijing Quanshijin Biotechnology Co., Ltd.; Annexin V PE/7AAD kit and PI/RNase staining buffer from Becton, Dickinson and Company in the United States; human FGF-3 Protein from R&D Systems in the United States, PD173074 (FGFR inhibitor) from MedChemExpress in the United States; and both primary and secondary antibodies from Abcam in the United States.

### 2.2. Cell Preparation

Human tongue squamous cell carcinoma SCC-9 cells were grown in Dulbecco's Modified Eagle Medium high-glucose medium with penicillin-streptomycin antibiotics and 10% FBS and grown at 37°C with 5% CO_2_. When cells reached 70% to 85% confluency, they were digested and passaged, and cells in the logarithmic growth phase were used for subsequent experiments.

### 2.3. Preparation of FGF3 Intervention

SCC-9 cells reaching 90% confluency were seeded at 5 × 10^4^ cells/mL in 96-well plates with complete medium (100 *μ*L/well or 5 × 10^3^ cells/well). After culturing at 37°C and 5% CO_2_ for 24 h to adhere to the well, the medium was discarded and four groups were set up: a blank control group and three other groups to which 100 *μ*L of FGF3 solution at different concentrations (10, 50, and 100 ng/ml) was added. Each group had 5 replicates and 3 collection time points (24 h, 48 h, and 72 h). A total of 100 *μ*L complete medium including 10 *μ*L of CCK-8 reagent was added to each well, and cells were incubated for 1 h. The optical density (OD) at 450 nm was measured using a microplate reader. To analyze our data, we calculated the survival rate of SCC-9 cells under the three different concentrations of FGF3 at the three different time points.

### 2.4. Groups and Interventions

In the control group, SCC-9 cells were cultured for 72 h. In the FGF3 intervention group, they were cultured for 72 h in medium with 100 ng/ml FGF3. In the FGFR inhibitor intervention group, they were cultured for 72 h in medium with 100 nM FGFR inhibitor PD173074.

### 2.5. Cell Proliferation Assay

SCC-9 cells were cultured in high-glucose medium solution containing FBS and penicillin-streptomycin antibiotics and tested in vitro. SCC-9 single-cell suspensions (5 × 10^4^ cells/mL) were inoculated in 96-well plates. Cells were placed in the incubator for 24 hours to allow for cell adhesion, and groups of cells were prepared as described above. A total of 100 *μ*L medium containing 10% CCK-8 solution was added to cells, cells were incubated for 1 h, and the OD at 450 nm was measured using a microplate reader. The survival rate of SCC-9 cells was calculated under different concentrations of FGF3 in the intervention group.

### 2.6. Cell Cycle Assay

Cells in each group were digested using trypsin and washed with phosphate-buffered saline (PBS). Cells were resuspended in 500 *μ*L of precooled PBS, added to 3.5 ml of precooled 80% ethanol, and were fixed at 4°C overnight. Cells were pelleted by centrifugation at 2000 rpm for 5 minutes. Supernatant was discarded, and cells were washed twice in PBS, with supernatant discarded each time. Cells were resuspended in 500 *μ*L of PI/RNase staining buffer, passed through a 200-mesh nylon to make a single-cell suspension, and incubated at 4°C for 30 minutes in the dark. A flow cytometer was used to detect red fluorescence at an excitation wavelength of 488 nm and measure light scattering. Cellular DNA content and light scattering were analyzed.

### 2.7. Apoptosis Assay

Cultured medium was aspirated, and adherent cells were washed twice in PBS, trypsinized, and centrifuged at 1000 rpm for 5 min. Supernatant was discarded, and cells were washed twice with precooled PBS, with supernatant discarded after each wash. To prepare single-cell suspensions, 500 *μ*L of 1 × binding buffer was added to cells, and suspensions were filtered through a 200-mesh sieve. A total of 5 *μ*L Annexin V-PE and 10 *μ*L 7-AAD was added to each group, and samples were mixed gently and placed in the dark at 4°C for 10 min. Apoptosis rates of SCC-9 cells were detected by flow cytometry after 30 min.

### 2.8. RT-PCR Detection of mRNA

RT-PCR was used to detect IRS1, PI3K (PIK3CA), AKT, BCL-2, and BAX genes in the blank, FGF3 intervention, and FGFR inhibitor intervention groups, with actin used as an internal reference. The primers used are shown in Table 1. The relative expression level of the target gene was expressed as 2^−*ΔΔ*Ct^.

### 2.9. Western Blot

After groups of cells were prepared as described above, cells were centrifuged, the supernatant was discarded, and cells were collected after washing with 5 mL of sterile PBS. Antibodies were used at a concentration of 1 : 1000. The total protein was extracted, denatured, separated with SDS-PAGE, and transferred onto membranes. Membranes were blocked and incubated overnight in primary antibody solution and then incubated in secondary antibody solution to obtain the expression of target proteins. Experiments were repeated three times, and the results were processed with ImageJ using *β*-actin as a positive control.

### 2.10. Statistical Analysis

Data were preprocessed in Excel, categorical variables were expressed as frequency (%), and continuous variables were expressed as means (with standard deviation (SD)) or medians (with interquartile range (IQR)). An *F* test was used to compare differences between multiple groups, and chi-square tests were used to analyze categorical data. A statistically significant level was set at 0.05. All statistical analyses were performed in SPSS software version 20.0.

## 3. Results

### 3.1. Determination of FGF3 Concentration and Time

An FGF3 concentration of 100 ng/ml for a time of 72 h was selected based on results of the SCC-9 cell growth curve and survival rate of SCC-9 cells (Figure 1).

### 3.2. Effects of FGF3 on the Proliferation of SCC-9 Cells

Results of the CCK-8 assay showed that the survival rates of cells in the control group, FGF3 intervention group, and FGFR inhibitor intervention group were 100.000% ± 4.026%, 136.330% ± 9.779%, and 83.199 ± 4.954%, respectively. Based on the comparison in the survival rate of cells between the FGF3 intervention group and control group and between FGFR inhibitor intervention group and the control group, we found that low expression of FGF3 inhibited the proliferation of tongue cancer cells (both *P* < 0.05). These results suggest that FGF3 promotes the proliferation of tongue cancer cells (Figure 2).

### 3.3. Effects of FGF3 on SCC-9 Cell Cycle and Apoptosis Rate

The effect of FGF3 on the SCC-9 cell cycle and apoptosis rate was assessed using flow cytometry. The ratio of cells in G0/G1 phase in the FGF3 intervention group was lower than that of the control group (*P* < 0.05), and the ratio of cells in G2/M phase was higher than that of the control group (*P* < 0.05). The ratio of cells in G0/G1 phase in the FGFR inhibitor intervention group was higher than that of the control group (*P* < 0.05), and the ratio of cells in G2/M phase was lower than that of the control group (*P* < 0.05) (Figure 3(a)). The apoptosis rate in the control group, FGF3 intervention group, and FGFR inhibitor intervention group were 5.867% ± 0.945%, 6.100% ± 0.624%, and 18.833% ± 1.242%, respectively. No significant difference was identified in the apoptosis rate of SCC-9 cells between the FGF3 intervention group and the control group (*P* > 0.05), while the apoptosis rate of SCC-9 cells in the FGFR inhibitor intervention group was significantly higher than that of the control group (*P* < 0.05). This data suggests that low expression of FGF3 promotes the apoptosis of tongue squamous cells and that FGF3 inhibits the apoptosis of SCC-9 (Figure 3(b)).

### 3.4. Activation of FGF3 on the PI3K/AKT Pathway of SCC-9

#### 3.4.1. RT-PCR Detection Results

Compared with the control group, the mRNA expression levels of IRS1, PI3K, and BCL-2 in the FGF3 intervention group increased (*P* < 0.05), BAX decreased (*P* < 0.05), and there was no significant difference in AKT. In the FGFR inhibitor intervention group, the mRNA expression levels of PI3K and BCL-2 decreased (*P* < 0.05), while BAX increased (*P* < 0.05), and there was no significant difference in IRS1 and AKT (Figure 4).

### 3.5. Western Blot Results

Compared with the control group, protein expression of IRS1, PI3K, and BCL-2 in the FGF3 intervention group increased (*P* < 0.05), and BAX expression decreased (*P* < 0.05). In the FGFR inhibitor intervention group, IRS1 protein expression decreased (*P* < 0.05), PI3K and BCL-2 protein levels showed a downward trend, and BAX protein expression increased (*P* < 0.05). While levels of p-AKT did not change, the expression of p-AKT protein showed a downward trend (Figure 5).

## 4. Discussion

Tongue cancer is prone to local recurrence and regional lymph node metastasis, with a high degree of malignancy and poor prognosis for patients. Understanding mechanisms for the proliferation and apoptosis of tongue cancer cells can guide prevention and treatment. The FGF family consists of 22 ligands. FGF11–14 are called intracellular FGFs, as they do not activate FGFRs and function independently of FGFRs. The remaining FGFs are dependent on FGFRs (FGFR1, FGFR2, FGFR3, and FGFR4) to exert their biological effects. The binding of ligands to receptors can promote receptor dimerization and activate downstream signaling pathways, including RAS/MAPK and FRS2/PI3K/AKT, among others [9–12]. FGF3 functions by binding to FGFR1 and FGFR2 receptors. FGFR inhibitors (PD173074) can effectively inhibit FGFR1–3 receptors, thereby blocking downstream effects of FGF3 [13].

Some studies have shown that FGF3 is involved in the proliferation and migration of malignant tumors. However, few studies have focused on FGF3 and the proliferation of oral squamous cell carcinoma. Both in vivo and in vitro studies from Zhang et al. showed that knockdown of FGF3 in colon cancer HT-29 cells significantly slowed down the migration of colon cancer cells compared with a control group. They observed that the tumor volume of FGF3 knockdown mice was significantly smaller than that of a control group. Further, knockdown of FGF3 was shown to inhibit colon tumor growth. In the present study, we overexpressed and inhibited FGF3 in tongue squamous cell carcinoma cells. Results from our functional experiments suggest that high expression levels of FGF3 promote tongue cancer proliferation, consistent with the role of FGF3 in other malignant tumors. Our data suggests that FGF3 promotes the proliferation of the tongue cancer cell line SCC-9.

A previous work in Huang et al. showed that in colon cancer HT-29 cells, when FGF3 was inhibited by a plasmid vector, the ratio of G0/G1 phase and G2/M phase was significantly changed, and more cells were blocked in the G2/M phase. Compared with the untransfected group, the number of cells remaining in S phase was significantly reduced. Our study showed that FGF3 also significantly changed the proportion of cells in the G0/G1 phase and G2/M phase. Compared to the control group, the ratio of cells in G0/G1 phase in the FGF3 intervention group was lower (*P* < 0.05), and the ratio of cells in G2/M phase was higher (*P* < 0.05). The ratio of cells in G0/G1 phase in the FGFR inhibitor intervention group was higher than that of the control group (*P* < 0.05), and the proportion of cells in G2/M phase was lower than that of the control group (*P* < 0.05). This data suggests that FGF3 is involved in regulating the cell cycle of tongue cancer SCC-9 cells.

Some studies have shown that the apoptosis rate of untreated colon cancer HT-29 cells is 0.22%, but following FGF3 inhibition, this rate becomes 3.88%, suggesting that inhibition of FGF3 can significantly promote tumor apoptosis. Our present study also showed that inhibition of FGF3 could increase tumor apoptosis. To clarify how FGF3 regulates tumor cell apoptosis, we further studied the IRS1/PI3K/AKT signaling pathway. Gene expression levels showed that mRNA expression increased for IRS1, PI3K, and BCL-2 in the FGF3 intervention group (*P* < 0.05). The expression level of BAX mRNA decreased (*P* < 0.05), and there was no significant difference in the expression level of AKT mRNA. Analyzing protein expression levels showed that IRS1, PI3K, and BCL-2 increased in the FGF3 intervention group (*P* < 0.05), and BAX protein expression levels decreased (*P* < 0.05). In the absence of changes in the total amount of AKT protein, p-AKT protein expression increased (*P* < 0.05), suggesting that FGF3 can promote phosphorylation of the AKT protein. Together, these results suggest that apoptosis may be regulated by the IRS1/PI3K/AKT signaling pathway. As a proangiogenic factor, FGFs is produced by tumor cells and macrophages or released from the extracellular matrix and acts in an autocrine or paracrine manner [14]. However, further research is required to determine involvement of FGF3 in the pathogenesis of tongue squamous cell carcinoma.

The results of this study show that FGF3 promotes the proliferation of tongue cancer SCC-9 cells and increases the proportion of cells in the G2/M phase. Inhibiting FGF3 can promote tumor apoptosis, and the mechanism may be through the IRS1/PI3K/AKT signaling pathway. FGF3 is involved in the occurrence, development, and pathogenic process of tongue cancer. These results provide a novel target for the precise treatment of tongue cancer with a mechanism of action that requires further study.

## Figures and Tables

**Figure 1:** Effects of fibroblast growth factor 3 (FGF3) intervention on the proliferation of squamous cell carcinoma SCC-9 cell line (SCC-9) cells at different time points (100×). Note: ∗ compared with FGF3 (0 ng/mL), *P* < 0.05; # compared with FGF3 (10 ng/mL), *P* < 0.05; & compared with FGF3 (50 ng/mL), *P* < 0.05. *n* = 3.

**Figure 2:** Cholecystokinin octapeptide (CCK-8) assay to determine effect of fibroblast growth factor 3 (FGF3) on the proliferation of squamous cell carcinoma SCC-9 cell line (SCC-9) cells (100x). Note: ∗ compared with control group, *P* < 0.05; *n* = 3.

**Figure 3:** Effect of fibroblast growth factor 3 (FGF3) on the cell cycle (a) and apoptosis rate (b) of squamous cell carcinoma SCC-9 cell line (SCC-9) cells measured by flow cytometry. Note: ∗ compared with control group, *P* < 0.05; *n* = 3.

**Figure 4:** Analysis of mRNA levels of each gene in cells of each group. Note: ∗ compared with control group, *P* < 0.05; *n* = 3.

**Figure 5:** Western blot detecting expression of different proteins in each group. Note: ∗compared with control group, *P* < 0.05; *n* = 3.

**Table 1:** List primers used for RT-PCR.

Genes	Primer sequence
AKT-F	GTCATCGAACGCACCTTCCAT
AKT-R	AGCTTCAGGTACTCAAACTCGT
PI3K-F	AGTAGGCAACCGTGAAGAAAAG
PI3K-R	GAGGTGAATTGAGGTCCCTAAGA
IRS1-F	CTGCACAACCGTGCTAAGG
IRS1-R	CGTCACCGTAGCTCAAGTCC
BAX-F	GCAAACTGGTGCTCAAGGC
BAX-R	GGCGTCCCAAAGTAGGAGA
BCL-2-F	CCGCGACTCCTGATTCATTG
BCL-2-R	ACAGCATGATCCTCTGTCAAGT
*β*-Actin-F	CATGTACGTTGCTATCCAGGC
*β*-Actin-R	CTCCTTAATGTCACGCACGAT

## Data Availability

The data used to support the findings of this study are available from the corresponding author upon request.
